# Prediction of Metal Ion Binding Sites of Transmembrane Proteins

**DOI:** 10.1155/2021/2327832

**Published:** 2021-10-22

**Authors:** Jing Qu, Sheng S. Yin, Han Wang

**Affiliations:** ^1^Systems Engineering Research Institute, Beijing, China; ^2^Institute of Computational Biology, School of Information Science and Technology, Northeast Normal University, Changchun, China

## Abstract

The metal ion binding of transmembrane proteins (TMPs) plays a fundamental role in biological processes, pharmaceutics, and medicine, but it is hard to extract enough TMP structures in experimental techniques to discover their binding mechanism comprehensively. To predict the metal ion binding sites for TMPs on a large scale, we present a simple and effective two-stage prediction method TMP-MIBS, to identify the corresponding binding residues using TMP sequences. At present, there is no specific research on the metal ion binding prediction of TMPs. Thereby, we compared our model with the published tools which do not distinguish TMPs from water-soluble proteins. The results in the independent verification dataset show that TMP-MIBS has superior performance. This paper explores the interaction mechanism between TMPs and metal ions, which is helpful to understand the structure and function of TMPs and is of great significance to further construct transport mechanisms and identify potential drug targets.

## 1. Introduction

Metal ions are vital to live organisms involving in various biological processes. They can enter cells to regulate the expression and activation of multiple biomolecules, participate in cell signal transduction, and complete various functions. For example, Ca^2+^ signaling is essential for T cell activation, autoantigen tolerance, differentiation, and development [1]. Mg^2+^ regulates ion channels' activity in cardiac cells, affecting the myocardium's electrical properties [2]. Zn^2+^ is a multitasking tool necessary to stimulate various enzyme activities [3] that lack and excess can cause central nervous system diseases [4, 5]. Also, other metal ions [6–10] perform their respective biological functions. Their homeostasis disorders involve neurodegenerative diseases, cardiovascular diseases, bone diseases, asthma, cancer, and diabetes [11]. Therefore, maintaining the correct levels of metal ions in the cytoplasm is essential for life and health.

As we know, metal ions cannot directly penetrate the cell membrane unless the transporter's assistance is on the cell membrane. According to the transport mode and spatial structure, the transporter protein can be roughly divided into channel and carrier proteins, all transmembrane proteins (TMPs). These particular proteins cross through the biomembranes by their transmembrane domains and exist therein whole life, constitute 15-30% of the genome [12]. TMPs, as the primary carrier of metal ions, participate in signal transduction, intracellular trafficking, and maintaining homeostasis [13, 14]. However, knowledge about the transport mechanism of metal ions that bind to proteins across membranes is still insufficient and varies for different metals. Exploring the TMPs' metal ion binding site (MIBs) provides a practical means to explore the ion selectivity and crucial abilities and even further construct the ion transport mechanism.

Experimental techniques such as AFM [15], MS [16], IMAC [17, 18], NMR [19], and X-ray crystallography [20] are comprehensive to identify the crystal structures of protein and characterize the binding sites in proteins. However, these techniques had not achieved large-scale application compared to the water-soluble proteins since the TMPs' folding, native structure, stability, and activity are reached only within the lipid bilayer [21]. With sequencing technology development, the time has come to study the work related to TMPs. Previous extensive research on water-soluble proteins has provided ideas in computational methods for use as reference. These methods, computation-based, reduce the cost to discover the potential MIBs that also have near-accurate predictions.

Over the last decade, computational methods have been made significant advances in identifying MIBs. Yang et al. combined two methods based on substructure and sequence (COACH [22]) to identify protein-ligand binding sites and achieved Matthews correlation coefficient (MCC) of 0.54. Zhao et al. present a 3D template-based metal site prediction (TEMSP [23]) to predict zinc binding sites and completed sensitivity of 0.86. Lin et al. used a fragment transformation method (MIB [24]) to predict twelve metal ion-binding sites with overall accuracy from 0.92 to 0.95. Yu et al. report a ligand-specific template-free predictor (TargetS [25]) for identifying protein-ligand binding sites that contain five metal ions overall MCC from 0.14 to 0.69. Hu et al. proposed a ligand-specific and template-based components approach (IonCom [26]) to predict 13 ions and achieved MCC from 0.14 to 0.69. Cao et al. [27] used only sequence information for multiple metals and yielded an overall accuracy from 0.62 to 0.84. Kumar [28] used the amino acid sequence information and machine learning approach to predict six metal ion binding sites' accuracy 0.86 to 0.87. Qiao and Xie developed a sequence-based ligand-specific predictor (MIonSite [29]) to predict 12 metal ion binding sites and completed MCC from 0.17 to 0.68. Haberal and Ogul [30] present deep learning architectures to predict metal binding of histidines (HIS) and cysteines (CYS) amino acids and acquire the precision 0.79 and recall 0.82.

Although the prediction of the binding site of metal ions and proteins has been fruitful, it cannot be directly applied to TMPs [31–34]. First of all, the above methods can be roughly summarized into structure-based and sequence-based. The former has better prediction performance, but the latter is more common. In the past, one of the impediments to this effort related to ion channels is that TMPs' structures have been notoriously difficult to obtain. Therefore, the performance of structure-based is limited in TMPs. Then, sequence-based methods of MIBs did not distinguish between TMPs and water-soluble proteins, while TMPs have significant conformational differences with those water-soluble proteins. Structurally, metal ions pass through the body of TMPs while they had never done so to any water-soluble protein. Functionally, water-soluble proteins cannot take on the responsibility of transporting metal ions inside and outside the membrane. Finally, TMPs have selective specificity for metal ions, which allows only a suitable size of metal ions to pass through. Therefore, ignoring the natures as mentioned above is incompatible with biological significance.

In this study, we proposed a metal-specific method for predicting the binding sites of the transmembrane protein and metal ions (TMP-MIBS) from protein sequence information. We selected five kinds of TMPs' specific structural or biochemical features: evolutionary information, physicochemical properties, solvent-accessible surface area, topology structure, and *Z*-coordinate features. TMP-MIBS was well trained against an up-to-date dataset collected from the PDBTM database. The sliding windows were introduced to build feature spaces, and random undersampling was utilized to tackle sample imbalance. The performance of the model is gradually improved through a two-stage learning process. In the first stage, metal ion binding sites of TMPs were identified. In the second stage, specific recognition models were constructed for the metal-specific. We have not yet found any tool specifically for binding site prediction about metal ion prediction and TMPs, so we compared ours with the published means for metal ions and general proteins. Our model achieves the best performance except for Ca^2+^. The work has culminated in a relatively effective tool for predicting metal binding sites without 3D structures. It has guiding significance for understanding and ultimately controlling the binding ability of metal ions and their application in drug and disease treatment in the future.

## 2. Materials and Methods

### 2.1. Datasets

The PDBTM [35] database (available at http://pdbtm.enzim.hu), which aims to collect all the TMPs from the protein structure database (PDB) and keep up to date with PDB, is the source of the data in this work. We screen protein data containing metal ion binding sites and parse sequences from the PDB file by applying the following criteria.

1. Only keep chains with residues that participate in binding metal ions when the proteins have more than one polypeptide chain
2. The length of the polypeptide chain is required to exceed 50 residues
3. Removing the protein sequences with sequence similarities greater than or equal to 40% by Cd-Hit [36]

Finally, there are 427 protein chains left as the experimental dataset. To evaluate the effectiveness of our model, we divide the training dataset and the independent verification dataset as listed in Table 1.

### 2.2. Feature Extraction

#### 2.2.1. Evolutionary Information

The sequence-based methods mainly rely on residue conservation analyses assuming that ligand binding residues are functionally important and should be conserved in the evolution [37–39]. By running the PSI-BLAST program on the server, iteratively searched the NR database three times and used 0.001 as the *E*-value cutoff of multiple sequence alignments to obtain evolution information of the protein sequence. We generated the position-specific scoring matrix (PSSM). The *L* residue's protein sequence generates an *L* × 20 matrix.

#### 2.2.2. Physicochemical Properties

Early studies in the prediction of transmembrane (TM) helices had widely used physicochemical properties (PCP) such as hydrophobicity analysis [40], the positive inside rule [41–43], and charge bias which are indeed valid. Besides, the residues binding with metal ions have many distinctive properties, such as electron-acceptor ability, positive charge, ion size, specific ligand affinity, varying valence state, and low or high spin configuration [44]. We collected the 553 physicochemical properties that influence the microenvironment of proteins. They were obtained from AAindex [45]. The protein sequence of the *L* residue generates an *L* × 553 matrix.

#### 2.2.3. Solvent-Accessible Surface Area

The solvent-accessible residues could be responsible for acquiring metal and may act as a potential metallochaperone to deliver metal to the TM region [46]. We calculate the relative solvent accessibility surface area (rASA) by MemBrain [47] for each residue to provide the residues' relative positions, which characterize TMPs' structure. The protein sequence of the *L* residue generates an *L* × 1 matrix.

#### 2.2.4. Topology Structure

Knowledge of the TM helices' presence and the exact location is essential for functional annotation and direct functional analysis. The prediction of topology structure (TOPO) serves to quickly obtain fundamental structural knowledge of TM proteins [48]. We used TMHMM-2.0 [49], which predicts the sequence's most probable location and orientation of transmembrane helices. The protein sequence of the *L* residue generates an *L* × 3 matrix.

#### 2.2.5. *Z*-Coordinate

The *Z*-coordinate (Zcoord) is defined as the residue's distance to the center of the membrane [50] and reflects the high correlation with the ligand binding and the protein-protein binding regions [51]. It implicitly contains information about TMPs' secondary structure, such as re-entrant helices, interfacial helices, a TM helix's tilt, and loop lengths. TOPCONS [52] was used to predict the Zcoord. The protein sequence of the *L* residue generates an *L* × 1 matrix.

### 2.3. Methods

#### 2.3.1. Outline

TMP-MIBS employs a two-stage learning process and an ensemble of models to improve prediction performance gradually. The obtained data were preprocessed and extracted the protein sequence and feature. All binding residues (the 24 kinds of metal ions) are predicted to identify the MIBs in the first stage. The second stage indicates the most probable location and binding probability of MIBs for seven classes which are K^+^, Ca^2+^, Na^+^, Zn^2+^, Mg^2+^, Hg^2+^, and others. We test two-stage models on the independent verification dataset to examine the performance of the model. More details on how our final model was built and trained are explained below.

#### 2.3.2. The First Stage of the Learning Process

When constructing the feature space is generated as the input of the first stage of the model, the sliding window strategy is used to intercept the amino acid fragments, and the random undersampling is introduced to extract some negative samples. Random forest (RF) is used as the prediction model and vote for binary class and selects the classification having the most votes. For a given protein sequence, the classifier outputs the exact conclusion that each residue is or is not a MIBs. This stage only predicted whether the residue would be binding with one in the 24 metal ions.

#### 2.3.3. The Second Stage of the Learning Process

The second stage learning process takes into account the ligand-specific. After the first model training stage, two prediction results, “1”and “0”, are output, corresponding to MIBs and non-MIBs. To further predict the binding of amino acid residues to metal ions, it is necessary to model the samples with the prediction result of “1” and enter the second stage of model learning. The second stage models the seven types of metal ions with the most significant number of sites, respectively. The OVR strategy in the multiclassification problem is adopted. Each time, the examples in one class are regarded as positive classes, and all other classes are taken as counterexamples. Finally, the seven classifiers for seven class metal ions output the probabilities for each residue binding residue in the given protein sequence.

### 2.4. Random Undersampling

Undersampling is a common technique among the existing technologies to overcome the sample imbalance problems. All the binding sites (positive samples) are kept, and the nonbinding sites (negative samples) as an original dataset *S* will generate a new set *S*′. The numbers are *N* times the positive samples (*N* takes an integer). We set the ratio parameter of positive and negative samples to 1 : 5, with the *N* design details explained in Section 3.4.

### 2.5. Sliding Windows

The structural state of a residue is determined not only by amino acid residue itself but also by neighboring residues. The interception of the neighbor residue length is critical to the description of the target residue. Underintroducing the information of neighbor residues is not conducive to distinguishing, but overintroducing may cause noise. The sliding window strategy is widely used to contemplate the influence of neighbor residues for the target residuals, located in the middle, and (*w* − 1)/2 adjacent residues are found on both sides ((*w*) size, being an odd number). Since the volume of metal ions is usually small, the optimal window length of metal ions should be smaller than that of the larger ligands, such as ATP and NAD ligands (17 in general) [53]. We computed and analyzed evaluation indicators for seven class metal ions to determine the optimal sliding window length.

### 2.6. Validation and Evaluation Metrics

Random 10-fold cross-validation was used to validate model and tuning parameters, which one set was used for testing, and the remaining sets were used for training. We randomly divided the dataset into ten sets. Repeat this process ten times, and the final score was obtained by averaging the performances. We used five evaluation measures to evaluate the generalization ability of the model, which are accuracy (ACC), specificity (SPE), sensitivity (SEN), Matthews correlation coefficient (MCC), and area under ROC curve (AUC), respectively [54–57]. The training dataset is used to fine-tune the proposed methods' parameters, and the independent test is used to test the methods.

(1) $$\begin{array}{c} \text{ACC}=\frac{\text{TP}+\text{TN}}{\text{TP}+\text{TN}+\text{FP}+\text{FN}}, \end{array}$$

(2) $$\begin{array}{c} \text{SPE}=\frac{\text{TN}}{\text{TN}+\text{FP}}, \end{array}$$

(3) $$\begin{array}{c} \text{SEN}=\frac{\text{TP}}{\text{TP}+\text{FN}}, \end{array}$$

(4) $$\begin{array}{c} \text{MCC}=\frac{\text{TP}\times \text{TN}-\text{FP}\times \text{FN}}{\left(\text{TP}+\text{FP}\right)\times \left(\text{TP}+\text{FN}\right)\times \left(\text{TN}+\text{FP}\right)\times \left(\text{TN}+\text{FN}\right)}, \end{array}$$

(5) $$\begin{array}{c} \text{AUC}=\frac{1}{2}\overset{m-1}{\underset{i=1}{\sum }}\left(x_{i+1}+x_{i}\right)∙\left(y_{i}+y_{i+1}\right), \end{array}$$

where TP, FP, TN, and FN represent true positive, false positive, true negative, and false negative.

## 3. Results and Discussion

### 3.1. Specific Binding of Metal Ions and Amino Acids

It is well known that ion channels are highly selective for controlling ions in and out, which can be reflected by combining different ions with amino acid residues [27]. We counted the frequency of amino acids and nonamino acids bound by metal ions to TMPs, as shown in Figure 1. Interestingly, (b) Ca^2+^, (d) Zn^2+^, (e) Mg^2+^, and (f) Hg^2+^have higher specificity when combined with residues than (a) K^+^ and (c) Na^+^. For Zn^2+^, it is more likely to connect with His (H), Cys (C), and Glu (E), which are polar amino acids. Mg^2+^ is more likely to bind ASP (D) and more minor to nonpolar amino acids. Hg^2+^ has the highest tendency to combine with amino acids containing the neutral R group, while Ca^2+^ has the most increased tendency to combine with acidic amino acids. Careful observation shows that metal ions are more likely to connect with hydrophilic amino acids than hydrophobic amino acids. The finding supports the hypothesis of solvent-accessible residues that act as a potential metallochaperone and participate in delivering metal to the TM region.

In addition, we can conclude that the difference in the binding frequency with amino acids reflects metal ions' physical and chemical properties. Metal ions under the main analogous group have similar chemical properties and also have similar selectivity. The selection of binding amino acid residues by metal ions of different main groups is also quite different.

### 3.2. Position Conservation of Amino Acids

We further studied the conservative position information of the above six MIBs by WebLogo [58], as shown in Figure 2. Sequences were intercepted in window length *L* of 21 as an example for each metal ion class to analyze. The relative size of letters (amino acids) indicates their occurrence frequency in the sequence. The larger the letter, the higher the frequency. According to the illustration, no matter the binding site or nonbinding site of K^+^ and Na^+^ is remarkable, reflecting the proximity of the two metal ion sites in sequence and structure. But the status of other metal ions (Ca^2+^, Zn^2+^, Mg^2+^, and Hg^2+^) makes the difference, which reflection of the binding site is remarkable, but the neighboring residues' contribution limits during the crucial process.

The degree of conservation demonstrates the importance of amino acids in evolution. A commonly cited approximation is that the more critical amino acids realize protein function, the less likely they will mutate. Thus, the conservation of amino acid residues is a good indicator of protein-metal ion binding. It was selected as the feature information to develop an effective identification model further.

### 3.3. Contribution of Features

The feature space contains five feature information, which we introduced in Section 2.2 for classifier learning. We compared the effects of adding different features on the results to verify the selected feature's validity.  Table 2 shows that five elements were verified by successively adding them into the classifier in the first stage of the learning process.

It can be seen from Table 2 that adding features in sequence from top to bottom plays a positive role for models in MCC indicators. On the one hand, the five characteristics selected in this experiment can better reflect the critical information of the TMP sequence and help the model identify the MIBs. On the other hand, five features are relatively independent and can play a more significant role when combined.

### 3.4. Random Undersampling Scheme

Exploring the ratio of binding and nonbinding residues is necessary to tackle the sample imbalance problem because too few negative samples will cause the loss of valuable information, and too many negative instances will increase the interference caused by redundant data.  Figure 3 depicts the change of evaluation indexes with the shift in positive and negative sample proportion in the first stage. We can see that the MCC value in the 10-fold cross-validation sets shows a decreasing trend with the ratio increase. In contrast, the MCC value on the independent set is fluctuant, but it increased in general. The ratio of negative sample sampling is the key to influence the final results. We used the proportion of positive and negative samples which is 1 : 5 to improve the model's overall performance.

### 3.5. Comparison with Other Machine Learning Methods over Cross-Validation

TMP-MIBS is based on the RF algorithm. This section compares the random forest with other machine learning methods on the training dataset, such as support vector machine (SVM), naïve Bayes, and AdaBoost. These methods have shown excellent performance in common classification problems. To obtain fair and objective experimental results, all models adopt the same dataset and preprocessing mechanism and finally get the test results shown in Table 3.

As shown in Table 3, the integration classes' performance is better than the others. Compare the two ensemble strategies AdaBoost and RF. The former adopts a boosting approach to ensemble base learners that adjust according to the previous one to generate prediction results serially, making the model susceptible to noise and outliers. Instead, the RF adopts a bagging strategy to make the base learner relatively independent and has no strong dependency. It can generate the prediction results in parallel, reduce outliers' influence on them, and have the natural advantage of solving the multidimensional unbalanced data. We further compared the prediction performance of different classifiers for each metal ion. The comparison similarly shows that the overall performance of the random forest classifier is optimal.

### 3.6. Comparison with Other Ligand-Specific Methods

To prove TMP-MIBS's robustness and effectiveness, we further tested the model on the independent testing dataset and compared it with two publicly available methods, including TargetS [25] and MIB [24]. The prediction performance was calculated based on the same dataset (Tables 1 and 4). For the TargetS method, a ligand-specific template-free protein-ligand binding site predictor used classifier ensemble and spatial clustering. It has five metal ligands that overlap with this study. We submitted the protein sequence into the webserver (http://www.csbio.sjtu.edu.cn/TargetS/) to obtain the predicted results and evaluate predictive performance. For the MIB method, which constructs metal ion binding templates for structural comparison between query proteins and templates and has four metal ligands identical to this study, we submitted and ran the MIB webserver (http://bioinfo.cmu.edu.tw/MIB/).

We observed that the performance of TMP-MIBS significantly outperforms the MIB on four metal ions. The average MCC value of Na^+^, Zn^2+^, and Hg^2+^ is about 16–39% higher than the TargetS. The results show that our model is superior to the available metal ion predictors, whether template-based or non-template-based methods. It can be inferred that the results largely depend on our input data rather than the complicated method. Although the number of TMPs sequences is increasing, it is still quite limited compared with non-TMPs. MIB and TargetS training models do not distinguish TMPs, so the models mainly learn the information of non-TMPs. The differences between the TMPs and non-TMPs are reflected in the secondary structure through sequence information and determine their tertiary conformation and function. TMP-MIBS focuses on TMPs, and the final results also confirm our efforts.

### 3.7. Metal Ion Binding Motif Analysis

A motif is an approximate sequence pattern that repeatedly occurs in a group of related sequences. It was used to reflect the protein's conservative information and discover novel information between different sequences. We tried to find out the motif within the metal ion binding domains to discover potential drug targets. The seven group metal ion binding domains were extracted for analysis.  Figure 4 shows the sequence logos of motifs for six metal ions and the 3D visualizations of their examples. Note that we stipulate the MEME outputs with ten motifs for each metal ion class and select the highest *E*-value for reporting.

From Figures 4(a)to 4(g), describe the logo of K^+^, Ca^2+^, Na^+^, Zn^2+^, Mg^2+^, Hg^2+^, and (g) other metal ions respectively. “*E*-value” is an estimate of the expected number of motifs with the given log-likelihood ratio (or higher). “Site Count” represents the number of sites contributing to the construction of the motif. “Width” represents the width of the motif. Sequences where each position is independent and letters are chosen according to the background letter frequencies. The red dashed box indicates the TMP-MIBS prediction site. The 3D visualization on the right is an example of the corresponding motif. “Protein” represents the PDB ID_Chain (domain).

The relative size of letters indicates their frequency in the sequence. It can be seen from the figure that the higher the letter, the more likely it is to become a binding site. Based on the extraction of motif sequence, we can predict the potential binding sites, which is helpful to understand further the biological significance involved in various biological processes.

## 4. Conclusions

Metal ions regulate almost all organisms' physiological cell functions, and their abnormal homeostasis usually leads to a variety of diseases and pathogenic states. They achieve homeostasis inside and outside the membrane and perform essential biological functions with TMPs' assistance. This study proposed an effective method to predict the binding residues of seven class metal ions in TMPs. We used the combination of conservative structure, physical and chemical properties, topological structure, solution accessibility, and *Z*-coordinate to apply the random forest algorithm to identify metal ion binding residues. These characteristics positively affected the prediction in essence. Test results show that TMP-MIBS has excellent performance for metal ion binding residues. This indicates that the sequential approach alone can achieve pleasant performance and demonstrates the importance of input data. With more and more sequence information obtained in the future, our model will show more excellent performance.

In the current work, a significant problem of TMB-MIBS is that predicting fewer MIBs on the protein sequence is still challenging. However, it can accurately predict more sites than existing tools because the imbalance of positive and negative samples is the unavoidable normal state of such problems. We will work to overcome this problem as the goal of the next phase.

## Figures and Tables

**Figure 1:** The amino acid binding frequency of six metal ions. The frequency of 20 kinds of amino acids on the binding site (blue) and nonbinding (red) was histogram. The abscissa represents the kinds of amino acids, and the ordinate represents the frequency (%); (a), (b), (c), (d), (e), and (f) represents K^+^, Ca^2+^, Na^+^, Zn^2+^, Mg^2+^, and Hg^2+^, respectively.

**Figure 2:** Position-specific conservation of amino acid residues. (a) K^+^, (b) Ca^2+^, (c) Na^+^, (d) Zn^2+^, (e) Mg^2+^, and (f) Hg^2+^.

**Figure 3:** The ratio of nonbinding residues and binding residues. (a) 10-fold cross-validation test. (b) Independent validation test.

**Figure 4:** Sequence logos of motif within the seven metal ion binding domains. (a) K^+^, (b) Ca^2+^, (c) Na^+^, (d) Zn^2+^, (e) Mg^2+^, (f) Hg^2+^, and (g) others.

**Table 1:** The training set and independent test set.

Category	Training dataset		Independent verification dataset	
Main	NProta	Nrecb	NProta	Nrecb
K^+^	63	202	6	17
Ca^2+^	78	388	10	51
Na^+^	54	223	7	46
Zn^2+^	52	241	5	26
Mg^2+^	64	209	10	27
Hg^2+^	8	83	3	25
Cu^2+^	14	54	2	9
W^6+^	13	56	1	4
Cd^2+^	8	31	2	10
Ni^2+^	10	28	3	9
Fe^3+^	7	19	0	0
Mn^2+^	7	32	0	0
Cu2	2	12	0	0
Rb^+^	4	18	0	0
Au^+^	2	13	0	0
Cs^+^	6	23	0	0
Pb^2+^	1	10	0	0
Fe^2+^	3	7	0	0
Pt^2+^	1	2	0	0
Sr^2+^	1	4	0	0
Li^+^	1	4	0	0
Co^2+^	3	4	0	0
Pr^3+^	1	3	0	0
Mo^6+^	1	1	0	0

NProta: number of protein entries; Nrecb: number of protein receptors bound with ions.

**Table 2:** The performance of different combinations of features.

Feature combination	ACC	SPE	SEN	MCC	AUC
PSSM	0.695	0.765	0.624	0.395	0.695
PSSM, PCP	0.75	0.801	0.7	0.504	0.75
PSSM, PCP, rASA	0.754	0.832	0.676	0.515	0.754
PSSM, PCP, rASA, Zcoord	0.755	0.834	0.675	0.516	0.755
PSSM, PCP, rASA, Zcoord, TOPO	0.766	0.861	0.67	0.542	0.766

**Table 3:** Comparison of RF with other classifiers.

Classifier	ACC	SPE	SEN	MCC	AUC
SVM	0.658	0.648	0.703	0.267	0.676
Naïve Bayes	0.767	0.775	0.73	0.409	0.752
AdaBoost	0.808	0.804	0.649	0.428	0.745
RF	0.795	0.808	0.73	0.447	0.769

**Table 4:** Comparison with publicly available methods.

Ligand	Method	ACC	SPE	SEN	MCC	AUC
K^+^	TMP-MIBS	0.981	1	0.118	0.34	0.559
Ca^2+^	MIB	0.942	0.943	0.342	0.067	0.643
	TargetS	0.997	0.999	0.471	0.494	0.735
	TMP-MIBS	0.908	0.998	0.196	0.398	0.597
Na^+^	TargetS	0.998	0.999	0.259	0.336	0.629
	TMP-MIBS	0.901	0.997	0.304	0.501	0.65
Zn^2+^	MIB	0.945	0.946	0.538	0.101	0.742
	TargetS	0.996	0.997	0.231	0.151	0.614
	TMP-MIBS	0.979	1	0.154	0.388	0.577
Mg^2+^	MIB	0.932	0.933	0.053	0	0.493
	TMP-MIBS	0.991	0.998	0.259	0.356	0.628
Hg^2+^	MIB	0.948	0.949	0.56	0.104	0.754
	TMP-MIBS	0.973	0.998	0.259	0.502	0.63
Others	TMP-MIBS	0.976	0.987	0.056	0.041	0.521

## Data Availability

TMP-MIBS's code and dataset are available at https://github.com/QuJing785464/TMP_MIBS.
